# Association between Immunohistochemistry Markers and Tumor Features and Their Diagnostic and Prognostic Values in Intrahepatic Cholangiocarcinoma

This article has been retracted.

**DOI:** 10.1155/2022/8367395

**Published:** 2022-04-28

**Authors:** Jiannan He, Cao Zhang, Qinye Shi, Fangping Bao, Xiang Pan, Yue Kuai, Jingjin Wu, Li Li, Ping Chen, Yian Huang, Jianhong Xu

**Affiliations:** ^1^Department of Anesthesiology, The Fourth Affiliated Hospital, Zhejiang University School of Medicine, Yiwu, Zhejiang, China; ^2^Department of Anesthesiology, The First Affiliated Hospital, Zhejiang University School of Medicine, Hangzhou, Zhejiang, China; ^3^Department of Colorectal Surgery and Oncology, Key Laboratory of Cancer Prevention and Intervention, The Second Affiliated Hospital, Zhejiang University School of Medicine, Hangzhou, Zhejiang, China; ^4^Department of Gastroenterology, The First Affiliated Hospital, Zhejiang University School of Medicine, Hangzhou, Zhejiang, China; ^5^Department of General Surgery, The Fourth Affiliated Hospital, Zhejiang University School of Medicine, Yiwu, Zhejiang, China

## Abstract

This study investigated the expression of some frequently used immunohistochemistry (IHC) markers. Besides, we evaluated their correlations with the clinical features and outcomes of intrahepatic cholangiocarcinoma (ICC). Patients who underwent surgical removal of the ICC tumors were followed up for 4 years. The paraffin-embedded sections were used to obtain different markers, including CK7, CK19, CK20, CDX2, Glypican3, Hepa1, Ki-67, Villin, and SATB1. Overall survival in relation to IHC marker expression patterns and other clinical characteristics was evaluated by Kaplan-Meier survival curve and log-rank test, followed by the Cox proportional hazard model (to evaluate the relationship between multiple factors and the overall postoperative survival). A total of 122 ICC patients (67 males and 55 females, averagely aged 57.75) were included in this study. There were 44 cases with vascular invasion, 46 cases with lymphatic metastasis, and 13 cases with distant metastasis. CK7 was negatively correlated with lymphatic metastasis; and in distant-metastasis cases, the positive ratio of SATB1 was lower. Interestingly, SATB1 expression indicated a poorer survival, while Villin expression was associated with a better survival. The COX regression analysis showed that female was a protective factor versus male, Villin expression was a strong protective factor, and Ki-67 expression was correlated with a poor survival. Together, IHC markers are associated with tumor features and postoperative survival, especially for SATB1 as a risk factor and Villin as a protective marker, and female ICC patients may have better survival than males.

## 1. Introduction

Intrahepatic cholangiocarcinoma (ICC), a rare primary malignant neoplasm, arises from intrahepatic biliary epithelia. It has a variable cholangiocytic differentiation. The incidence and mortality of ICCs have increased in recent years, and prognosis of ICC patients is poor. Currently, there have been very few recognized tumor markers for ICC but great needs to mine novel markers as diagnostic, prognostic, and therapeutic targets [1]. Immunohistochemistry (IHC) was used to study ICC carcinogenesis [2]. For example, hepatocellular progenitor cells label with CD56, CK7, SALL4, Okt4, CRP, and CK19. The large duct ICC does not express CD56 but generates S100P. The novel pancreatic cancer biomarkers TBX4, HSP60, and DJ-1 are also overexpressed in ICC tumors but with a relatively lower expression level in pancreatic ductal adenocarcinomas [3, 4]. Histologic features of the CK family, intestinal-specific transcription factors (e.g., CDX2), Glypican3, and SATB1 have also been used in recognizing ICC [5–8]. However, the prognostic values of these frequently used IHC markers have been largely unknown. Besides, we have previously noticed Villin (an actin modulator in the regulation of cell structure/plasticity and a polarity associated marker which may participate in colorectal micropapillary carcinoma, breast cancer, cholestasis, and pathology in hepatocyte [9–11]) was highly expressed in most of ICC cases. It is reasonable to hypothesize that some important ICC-related proteins have links to the later survival. The contribution of the present study was to investigate the expression of some frequently used IHC markers and assess their correlations with the clinical features and outcomes. In particular, we found some factors (Villin and STAB1) have significant prognostic values.

## 2. Materials and Methods

### 2.1. Study Design

This retrospective study collected the data of patients who underwent surgical removal of the ICC tumors and were followed up for 4 years. All included patients were determined to perform surgical findings. Only ICC primary cases were included, and patients with hilar, extrahepatic cholangiocarcinoma, purely intraductal neoplasms, invasive carcinomas from mucinous cystic neoplasms, and combined hepatocellular cholangiocarcinoma were excluded. Besides, individuals without surgical samples were also excluded. For each included case, clinical data including the basic demographic information and tumor characteristics were recorded. During the follow-up (at most 4 years), the survival status and period were recorded if a patient was contacted.

### 2.2. Immunohistochemistry

IHC staining was performed by the pathology department of our hospital according to the doctor's order. The 5 *μ*m paraffin-embedded tumor-tissue sections of 122 patients were used to obtain different markers, including CK7, CK19, CK20, CDX2, Glypican3, Hepa1, Ki-67 (%), Villin, and SATB1. Briefly, sections were deparaffinized and rehydrated. After boiling (antigen retrieval), sections were treated by methanol containing 3% hydrogen peroxide. Next, they were incubated with the primary antibodies (at 4°C overnight), the secondary antibodies (2 hours), and then 1 hour with the avidin–biotin–peroxidase, followed by DAB staining and hematoxylin re-dyeing. The expression level of each tumor marker was measured as negative (-), mild positive (+), moderate positive (++), or strong positive (+++) staining, and the low-expression markers in ICC were labeled negative (-) or positive (+).

### 2.3. Statistical Analysis

Data are expressed as numbers with proportions (%) or mean with SD. The differences in values derived from categorical variables were compared using the Chi-squared test or Fisher's exact test. The student's *t*-test or Mann–Whitney *U* test was applied for comparison between two groups of continuous variables; one-way ANOVA was used for three or four groups. The association of tumor biomarkers with the clinicopathological characteristics of IHCC patients was evaluated with Chi-squared or Fisher's exact test as appropriate. Overall survival in relation to IHC marker expression patterns and other clinical characteristics was evaluated by Kaplan-Meier survival curve and log-rank test. To assess the connection between numerous covariates and overall postoperative survival, the Cox proportional hazard model was utilized. The univariate analysis indicated statistically significant prognostic variables, which were then incorporated in the multivariate analysis. A *P* value < 0.05 was considered statistically significant.

## 3. Results

### 3.1. Demographic and Clinical Characteristics of Enrolled Patients

A total of 122 ICC patients (67 males and 55 females, averagely aged 57.75) were included in this study. As Table 1 shows, there were 64 tumors in the left outer lobe, one tumor in the left inner lobe, 48 tumors in the right anterior lobe, 8 tumors in the right posterior lobe, and 8 tumors in the caudate lobe. In aspect of tumor number, there were 92 cases with a single lesion, 3 cases with 2 tumors, and 22 cases with three or more tumors. In addition, there were 44 cases with vascular invasion, 46 cases with lymphatic metastasis, and 13 cases with distant metastasis. The pathological outcome showed that the mean diameter (maximum diameter of each tumor) was 5.58 ± 2.82 cm, and the average Ki-67 expression level was 44%.

### 3.2. Association between IHC Markers and ICC Tumor Features

The typical expression images of Villin, SATB1, Ki-67, Glypican3, CK7, CK20, CK19, and Hepa1 were presented in Figure 1. Among all IHC markers, CK7 was found negatively correlated with lymphatic metastasis (*P* < 0.05) (Table 2). As the expression of CK7 increased, the ratio of lymphatic metastasis decreased accordingly. Similarly, in distant-metastasis cases, the positive ratio of SATB1 was lower than metastasis negative cases (*P* < 0.05). Moreover, CK20 expression had a link to the tumor number, that the group with three or more tumors had all the +++ cases, and single-tumor cases had relatively lower expression of CK20 (*P* < 0.01). Together, IHC markers, including CK7, CK20, and SATB1, were associated with ICC tumor features.

### 3.3. Factors Associated with Postoperative Survival

Further, all available features, especially the IHC markers, were assessed about the prognostic values. Using the KM survival analysis, we noticed a significant association between postoperative survival and the expression of SATB1 and Villin (Figures 2(a) and 2(b)). Interestingly, SATB1 expression indicated a poorer survival (log rank *P* = 0.04) (Figure 2(a)). The medians survival time of the SATB1 negative cohort was 347 days (95% CI 188.240 to 505.760 days), and that of the SATB1 positive was 122 days (95% CI 74.941 to169.059 days). In contrast, the positive expression of Villin implied a better survival (log rank *P* = 0.002), in particular the ++ subgroup (Figure 2(b)). The medians survival periods of Villin -, +, ++, and +++ groups were 121 (95% CI 79.163 to 162.837), 156 (95% CI 71.458 to 240.542), 299 (95% CI 0.000 to 831.911), and 206 (95% CI 110.251 to 237.749) days, respectively. Next, the COX regression analysis of potential survival-associated factors was performed. Finally, the included factors were presented in Table 3. Among demographic characteristics, the influence of gender on postoperative survival was noticed, that female is a protective factor versus male. In consistency with the KM survival analysis, Villin expression was a strong protective factor. And as expected, Ki-67 expression was correlated with a poor survival. No statistical significances were found in other IHC markers. Together, female ICC patients may have better postoperative survival, and the IHC markers of tumor samples including Ki-67, SATB1, and Villin have prognostic values.

## 4. Discussion

In this work, we have three main findings: (1) IHC markers (CK7, CK20, and SATB1) are associated with ICC tumor features (including tumor number and metastasis), which suggested that these proteins may participate in the development of ICC; (2) female ICC patients may have better postoperative survival; (3) for ICC survival, Ki67 and SATB1 are risk IHC markers, and Villin is beneficial marker. To our best knowledge, these findings were discovered for the first time, and no similar results have been reported. Taking the gender advantage of females, for example, known risk factors of ICC specific mortality included liver fibrosis, vascular invasion, lymph node metastasis, comorbidities (liver diseases, ulcer, diabetes, etc.), resection margin in the surgery, and some preoperative inflammatory biomarkers in blood [12–16]; but there have no studies showing that females outperform males in postoperative ICC survival. This may be due to a lower level of inflammatory and liver disease severity in females.

Commonly, metastasis is a result of polarity weakening and epithelial-mesenchymal transition (EMT) [17–19]. CK7 is a type-II cytokeratin. It specifically expressed in the simple epithelia lining the cavities of the internal organs and in the gland ducts and blood vessels. CK7 has a diagnostic and prognostic value in lung carcinoma and hormophobe renal cell carcinoma [20–22]. In line, we found CK7 is negatively correlated with lymphatic metastasis in ICC for the first time, and this finding implied that assessment of CK7 in ICC tumor samples may provide information about the current clinical status and even subsequent progression.

SATB1 (a matrix protein binding nuclear matrix) is an oncogenic driver in most of carcinomas (including head and neck squamous cell carcinoma, nasopharyngeal carcinoma, and lung adenocarcinoma) [23–27]. Its role in ICC is largely unknown. Interestingly, we found SATB1 is negatively correlated with distant metastasis but positively with a poor prognosis. This may be attributable to a small number (and ratio) of distant metastasis cases in the whole pool (only 5 cases). Overall, it is a risk factor to survival, especially towards the patients without a distant metastasis. Consistently, it is a carcinogenic factor in our result and published studies (with an impact on EMT and metastasis [28, 29]), and the prognostic significance of SATB1 expression should be paid attention in ICC treatment.

Villin family may play a role in actin binding and structural constituent of cytoskeleton. Villin is a surface-related glycoprotein. It has been believed reverse-polarity biomarker in colorectal micropapillary carcinoma. Previously, it was reported that SATB2-and-CK20/Villin dual stain is effective to differentiate colorectal carcinomas [30–32]. In colorectal carcinomas, Villin plays an antiapoptotic role. However, its cleaved NH2-terminal can regulate epithelial cell extrusion from the villus tips by inducing apoptosis [33, 34]. However, its precise role in carcinogenesis has yet to be determined. Villin expression may be a protective factor for ICC survival, according to the results presented here. In support of this, it was discovered that when the intestinal epithelium is damaged, Villin targets F-actin and ensures microvillus depolarization. [35]. In addition, Villin expression is frequently lost in poorly differentiated colon cancer [36, 37]. These data indicate Villin may inhibit EMT and metastasis and play an antitumor role in colorectal cancers, and it is reasonable to believe it has a similar effect in ICC.

Still, there are some limitations in this study. For the limited sample size, the total cases of lymphatic and distant metastasis are small, and the statistical significance about metastasis-related results is still to be confirmed. We have only observed RFS but documented no data about the overall survival; hence, the influence of prophylaxis on the long-time survival is still to be assessed. Moreover, the diagnostic roles of STAB1, CKs, and Villin are not clear in this study given that no data of normal tissue were available for comparison.

## 5. Conclusions

In conclusion, IHC markers are linked to ICC tumor characteristics and postoperative survival, particularly SATB1 as a risk factor and Villin as a protective sign, and female ICC patients may outlive men.

## Figures and Tables

**Figure 1:** The typical expression images of Villin (a), SATB1 (b), Ki-67 (c), Glypican3 (d), CK7 (e), CK20 (f), CK19 (g), and Hepa1 (h).

**Figure 2:** The postoperative survival curves showing the risk marker SATB1 (a) and the protective marker Villin (b), and the female ICC patients have a better survival than females.

**(a):** 

Characteristics	Case number	%
Total cases	121	100%
Gender		
Male	67	54.9
Female	55	45.1
Tumor location (lobe)		
Left outer	64	52.5
Left inner	1	0.8
Right anterior	48	39.3
Right posterior	8	6.6
Caudate	8	6.6
Tumor number		
1	92	75.4
2	3	2.5
≥3	22	18.0
Vascular invasion		
No	78	63.9
Yes	44	36.1
Pathological differentiation		
Low	1	0.8
Medium	18	14.8
High	5	4.1
Lymphatic metastasis		
No	76	62.3
Yes	46	37.7
Distant metastasis		
No	109	89.3
Yes	13	10.7

**(b):** 

	N	Mean	SD
Age (years)	122	57.75	9.70
Maximum diameter (cm)	116	5.58	2.82
Ki-67 level	111	44%	24%

**Table 2:** Association between IHC markers and ICC tumor features.

Features	Markers	Expression level				*X* ^2^	*P* value
	CK7	—	**+**	**++**	**+++**	8.958	0.030
Lymphatic metastasis							
No		2	20	16	39		
Yes		4	7	3	31		
	SATB1	**—**	**+**			5.828	0.016
Distant metastasis							
No		6	35				
Yes		3	2				
	CK20	—	+	++	+++	19.776	0.003
Tumor number							
1		85	4	2	0		
2		3	0	0	0		
≥3		15	4	0	3		

**Table 3:** COX regression of postoperative survival using features of gender, Ki-67, and Villlin.

		B	SE	Wald	*P* value
Gender	Female vs. male	-1.465	0.474	9.541	0.002
Ki-67		1.836	0.818	5.037	0.025
Villin				13.917	0.003
	+ vs. -	-1.325	0.641	4.27	0.039
	++ vs. -	-2.885	0.82	12.377	<0.001
	+++ vs. -	-1.83	0.58	9.966	0.002

## Data Availability

The data used to support the findings of this study are included within the article.
